RETRACTED

# Diversity of Rotavirus Strains among Children with Acute Diarrhea in Karachi, Pakistan

**DOI:** 10.1155/2022/5231910

**Published:** 2022-04-23

**Authors:** Nain Tarra Bukhari, Gulnaz Parveen, Pir Asmat Ali, Amtul Sami, Yasmeen Lashari, Naila Mukhtar, Raisa Bano, Nargis Haider, Atiya Hussain Khowaja, Shahana Urooj Kazmi

**Affiliations:** ^1^Clinical Laboratory Sciences, Women University, Swabi, Pakistan; ^2^Department of Botany, Women University, Swabi, Pakistan; ^3^Department of Zoology, Women University, Swabi, Pakistan; ^4^Department of Microbiology and Molecular Biotechnology, Women University, Swabi, Pakistan; ^5^Department of Pathology, Bolan Medical College, Quetta, Pakistan; ^6^Department of Botany, University of Okara, Pakistan; ^7^Department of Public Health & Bioinformatics, Women University, Swabi, Pakistan; ^8^Department of Physiology, Bolan Medical College, Quetta, Pakistan; ^9^Agha Khan Medical University and Hospital, Karachi, Pakistan

## Abstract

One of the common viral pathogens in infectious diarrhea is *Rotavirus*; in developing countries, it is a primary cause of deaths in children less than five years of age. This study was planned to find out the etiologic agents of acute watery diarrhea. In this study, 1465 stool samples were analyzed with the symptoms of acute diarrhea. Demographic data analysis showed no. of episodes of diarrhea, vomiting, and fever. All samples were checked by ELISA technique for the presence of *Rotavirus* circulating strains. More than 6% patients were found to be positive with Rotavirus. Common *Rotavirus* genotypes, including G2P4, G2P6, G3P4, G8P4, G8P6, G9P4, and G10P4, were detected in patients through RT-PCR. This study concluded that detection of rotavirus strain diversity and management of diarrheal patients may identify assortment of emerging strains and reduce emergence of antimicrobial resistance and repeated episodes of diarrhea, which may also help to avoid and manage the essential nutrients lost leading to malnutrition and stunted growth, as well as to reduce high mortality rate in young children less than five years.

## 1. Introduction

*Rotavirus* is considered the major cause of severe gastroenteritis ranges from asymptomatic self-limiting watery diarrhea to life threatening infection in children worldwide. Malnutrition and stunted growth can occur if mismanaged in symptomatic cases ([1] [2]). Among these reported cases, 30% etiological agent are bacterial, viral, or parasitic [3]. Recently, 40-50% severe cases of infantile watery diarrhea are attributed to *Rotavirus* worldwide causing 600,000 deaths per year in African and Asian countries [4]. In a WHO 2015 report, 1.7 billion reported cases accounts 9% cumulative infantile deaths resulting in elevated health budget. According to earlier studies, 5.2 million bacterial, etiological agents along with 2.5 million parasitic and 30.9 million viruses cause diarrheal episodes [5]. In Pakistan due to multiple and recurrent diarrheal episodes > 150,000, deaths occur annually, leading infants towards malnutrition and retarded growth [6]. Almost 35%-50% of infected infants were between 1 and 2 years of age bracket [7]. Similarly, 2.5% cases were moderate in severity which progressed to life-threatening situation and were from low-socioeconomic settings, and the numbers of rotavirus cases were high where no health care facility was available [8]. The seasonal variation marker indicated that infection persists throughout the year having no correlation with rainy season while raise in no. of cases was reported in dry season. *Rotaviruses* in Pakistan are highlighted recently as an important nonbacterial etiological agent in young children [9]. Electron microscopy was only a tool to detect the virus, but recently, more advance techniques like enzyme-linked immunosorbent assay (ELISA) or latex agglutination rapid system and PCR method are in routine use to avoid blind therapy and emergence of MDR pathogens [10].

RETRACTED

The study was designed based on reports that in Pakistan after every minute a child dies due to diarrhea [11]. It is reported that 140,000 young population under five got *Rotavirus* infection, resulting, so leading them to malnutrition and stunted growth. This serious issue of high morbidity and mortality warrants investigation [12]. The aims and objectives of this present study are molecular identification of prevalent pathogenic strains of viral etiological agent, i.e., *Rotavirus*VP4, P8, P4, P6, P9, P10, and P11 and *Rotavirus* VP7, G8, G1, G2, G4, G3, and G9 by a PCR method using specific primer sets.

## 2. Material and Method

In this study, 1465 stool samples of acute watery diarrhea in premarked containers in duplicate in cold storage were collected from NICH and Civil Hospital Karachi and transported within 24 hours to central lab. Patients with complaint of acute watery diarrhea were included in the age bracket of 4 weeks to <5 years while those having other morbid conditions or bloody diarrhea were excluded and informed consent was taken. The questionnaire was designed to focus the parameters like No. of episode of diarrhea, fever, and vomiting.

### 2.1. Detection of *Rotavirus* by Sandwich ELISA

To detect the group-specific antigen, polyclonal antibody attached to wells in a sandwich enzyme immunoassay was used. The presence of rotavirus antigen was compared to color intensity above the cutoff value in the sample by adding 1-gram sample in 1 : 100 dilutions.

RETRACTED

### 2.2. Procedure of ELISA

*Rotavirus* antigen was detected by an ELISA kit method. Diluent buffer was added in 1 : 11 ratio whereas wash buffer and distilled water in 1 : 10 were made in test tubes. 100 *μ*l of diluted stool sample was taken. 100 *μ*l conjugate was added in assigned wells along with positive and negative controls. 60 minutes incubation at room temperature. Washing with diluted buffer 300 *μ*l. 15 minutes' incubation in dark chamber after addition of 100 *μ*l of substrate finally added 50 *μ*l of stop solution, ELISA plate reader at 450 nm for results.

### 2.3. Genotyping of *Rota* Isolates

*Rotavirus* genotyping was carried out using primer sets against capsid protein VP4 and VP7 coding genes from *Rotavirus* genomic RNAs (Tables 1 and 2). PCR mix contains a total volume of 50 *μ*l by adding 50 *μ*l of PCR mix, Invitrogen kit. Add 5 *μ*l of cDNA. Briefly spin before transfer to the thermocycler. First, cycle for 94°C for 2 min followed by 94°C, 50°C, and 72°C for 1 min in 35 cycles then for 7 minutes in 72 cycles followed by15°C on hold. Second round PCR mix consists of 5 *μ*l of the abovementioned amplified products in 50 *μ*l of master mix in microcentrifuge tubes, before transfer to the thermocycler.

At 100 mA *Rotavirus* genomic RNAs polyacrylamide gel by electrophoresis was detected in tank with buffer for 30 min. The migration of individual RNA genome segments was studied and compared with marker genome segments.

### 2.4. RT-PCR

Reverse transcriptase PCR was performed by taking genomic RNA 1 *μ*g in 25 *μ*l of RNase inhibitor (20 U of RNase out and DNA polymerase containing distilled water). At 50°C for 60 min, the process for reverse transcription was performed in a heating chamber. The termination of reaction was at 85°C for 5 min. Cooling of mix, 2 U of RNase H in 1 *μ*l followed by incubation 20 min at 37°C. 50-*μ*l processed for PCR containing 2.0 *μ*l of the RT-PCR products. Amplification buffer 5 *μ*l, 1.5 *μ*l of forward and reverse primer each adding, 2.5 U DNA polymerase. Denaturation of Template (94°C, 2 min), 30 cycles of PCR were set. PCR cycle set for denaturation step (94°C for 30 s), annealing (55°C for 30 s), and extension (68°C for 3 min for gene 4 and for 2 min for gene 6). Additional incubation (72°C, 7 min) followed by PCR. PCR purification kit (Qiagen) to collect purified DNA. By using RT-PCR as templates, VP4 and VP6 gene sequences were determined.

## 3. Result and Discussion

The current study found that many diversified strains of human *Rotavirus* are circulating in the community of Karachi as population belongs to nearby rural areas, where human interaction with animals makes it possible for the assortment for human and animal strains and emergence of new strains.

RETRACTED

In the present study, a prevalence of 6% (Figure 1) RVA in diarrheal cases from Pakistan was not too high as compared to those of other reported studies, but it is in correlation with reports that say *Rotavirus* infection prevalence rate in Eastern countries reported 40.5%-60.5% [13]. Similarly, 30%-56% prevalence was reported in Far East countries. A report from Karachi, Pakistan, a prevalence of RVA infections a little higher at 17% was noted which is probably due to the fact that we included patients with acute illness rather than advanced stage [14]. In Karachi, during the years from 2005 to 2007, different strains of *Rotavirus* in stool samples of children under five years of age—i.e., G9P8, G1P8, and G1P4, were of prime importance in addition to G2P4 (6%), G4P6, G9P6, and G9P4, whereas 2.4% mixed infection caused by more than one strain was also identified [13, 15].

In another study from Pakistan, G1P8, G2P4, G1P6, G9P8, G9P6, G12P6, G6P1, and mix infection with other pathogens were reported as causative etiological agents. These findings are indicative that RV genotype prevalence can be in various combinations and seasonal variation does not affect the prevalence of infection (Figure 2). Rotavirus genotypes G1P4, G1P6, G4P6, G9P4, G12P6, and G6P4 isolated from animals can have recurrent episodes of appearance or disappearance periodically. Our current study also highlighted that RT-PCR sometime does not detect false ELISA positive RV strains (due to multiple reasons like mutations in the genome, diminished viral load, or loss of viral antigenic sites during preservation) or there could be false positive ELISA results [15]. In present study, the data analysis of sick children showed that only 9.5% patients were found vaccinated and 90.5% children did not get vaccine against common diseases (Table 3). Similar results were obtained from.

In *Rotavirus* infection due to assortment of genes, several G types (G2, G3, G8, G9, and G10) and circulating P-types are a cause of mix infection in a single patient in multiple cases [16]. It is also reported in this study that 1.63% mixed VP7 infections: G1G2P4, G2G9P4, G2G9P6, and G2G9P8, were recorded in positive cases (Figure 3). A similar finding with 2.4% prevalence rate in Pakistan was also reported by Ali et al., [17]. Similarly, in South Korea, prevalence was reported mixed infections of 10% and 15% with interspecies transmission [18]. By using primer set against outer G and P antigen, molecular identification was done by visualizing bands of specific Bp on gel images which indicated the *Rotavirus* subtypes G2P4, G10P4, G9P4, and G3P4 (Figures 4 and 5).

RETRACTED

Pathogenesis might be the result of several assortments of human and animal strain resulting in origin of G11; however, from Pakistan, most of the focus was on VP7 and VP4 genotyping studies from different cities [19, 20]. It is reported that presence of animal origion RV strain among Pakistani patient is a result of interaction between humans and their livestock and reassortment of genes resulting new strains [19, 20]

In this study, it is noted that the presence of new mix strains of *Rotavirus* was detected in our population beside common circulating strains around the Globe. *Rotavirus* genotypes which were detected in our patients were G10P4, G2P4, G2P6, G3P4, G8P4, G8P6, and G9P4.

## 4. Conclusions

Spectrum of etiological agents is involved in diarrhea which is a huge health burden worldwide as well in Pakistan. The data of the current study indicate that by conducting prevalence studies and identifying risk factors disease can be timely prevented or managed. Thus, morbidity and high mortality in infants can be reduced. This issue warrants broad-spectrum investigation.

## Figures and Tables

**Figure 1:** Overall pathogen distribution.

**Figure 2:** Seasonal variation of rotavirus.

**Figure 3:** Rotavirus subtypes.

**Figure 4:** Rotavirus genotypes showing gene expression of VP–7 and VP–4 capsid protein coding genes.

**Figure 5:** Rotavirus genotypes VP–7 and VP–4 and primers for nonspecific protein expression genes.

**Table 1:** *Rotavirus* VP7 primer list.

Primer	Human sequence (5′-3′)	Position (nt)	Strain (genotype)	References
aAT8	GTCACACCATTTGTAAATTCG	178-198	69 M (G8) 885 bp	[21]
aBT1	CAAGTACTCAAATCAATGATGG	314-335	Wa (G1) 749 bp	[21]
aCT2	CAATGATATTAACACATTTTCTGTG	411-435	DS-1 (G2) 652 bp	
aDT4	CGTTTCTGGTGAGGAGTTG	480-498	ST-3 (G4) 583 bp	
aET3 mG3	CGTTTGAAGAAGTTGCAACAG ACGAACTCAACACGAGAGG	689-709 250-269	P 374 bp (G3) 682 bp	[22]
aFT9 mG9	CTAGATGTAACTACAACTAC CTTGATGTGACTAYAAATAC	757-776 757-776	W161 (G9) 306 bp 179 bp	[22]

**Table 2:** *Rotavirus* VP4 primer list.

Primer	Human sequence (5′-3′)	Position (nt)	Strain genotype	References
1T-1 1T-1D dP [9]	ACTTGGATAACGTGC TCTACTGGRTTRACNTGC	339-356 339-356	KU P8 P8	[21]
2T-1	CTATTGTTAGAGGTTAGAGTC	474-494	RV5 P4	
3T-1	TGTTGATTAGTTGGATTCAA	259-278	1076 P6	[22]
4T-1	TGAGACATGCAATTGGAC	385-402	K8 P9	[21]
5T-1	ATCATAGTTAGTAGTCGG	575-594	69M P10	[21]
mP11	GTAAACATCCAGAATGTG	305-323	MC435 P11 312 bp	[21]

**Table 3:** Vaccination status.

Vaccinated	No. of children (*n*)	%
Yes	139	9.5
No	1326	90.5
Total	1465	100.0

## Data Availability

Data can be provided on demand.
